# Nanoparticle albumin-bound paclitaxel as neoadjuvant chemotherapy of breast cancer: a systematic review and meta-analysis

**DOI:** 10.18632/oncotarget.14477

**Published:** 2017-01-03

**Authors:** Yu Zong, Jiayi Wu, Kunwei Shen

**Affiliations:** ^1^ Comprehensive Breast Health Center, Shanghai Ruijin Hospital affiliated to Shanghai Jiaotong University School of Medicine, Shanghai, China

**Keywords:** breast cancer, neoadjuvant, nab-paclitaxel, pathological complete response, toxicity

## Abstract

**Background:**

The value of nanoparticle albumin-bound paclitaxel (nab-paclitaxel) in neoadjuvant systemic therapy for breast cancer remains uncertain.

**Methods:**

Both electronic databases and proceedings of oncologic meetings were included in systematic literature search. Pooled rates of pathological complete response (pCR), odds ratios (ORs) and 95% confidence intervals (CIs) were calculated using fixed-effect or random-effect model to determine the effect of neoadjuvant nab-paclitaxel.

**Results:**

Twenty-one studies with 2357 patients were included, 3 of which were randomized clinical trials. The aggregate pCR(ypT0/is ypN0) rate was 32% (95% CI 25-38%) in unselected breast cancer patients and variated in different subtypes. Within randomized clinical trials, the probability of achieving pCR was significantly higher in the nab-paclitaxel group than in the conventional taxanes group (OR = 1.383, 95%CI 1.141-1.676, *p* = 0.001). For non-hematological toxic effect, any grade and grade 3-4 peripheral sensory neuropathy occurred more frequently with nab-paclitaxel compared to paclitaxel (any grade, OR = 2.090, 95%CI 1.016-4.302, *p* = 0.045; grade3-4, OR = 3.766, 95%CI 2.324-6.100, *p* < 0.001). Hypersensitivity was more common with paclitaxel than nab-paclitaxel at any grade and grade 3-4.

**Conclusion:**

nab-paclitaxel is an effective cytotoxic drug in neoadjuvant treatment of breast cancer, especially for aggressive tumors in terms of pCR. Exchange of nab-paclitaxel for conventional taxanes could significantly improve pCR rate with reasonable toxicities.

## INTRODUCTION

Breast cancer is the most common malignancy in women worldwide, and one of the leading causes of cancer death [1]. In routine clinical practice, neoadjuvant systemic therapy (NST) has become a widely accepted choice to treat patients with operable and locally advanced breast cancer [2]. Patients attained pathologic complete response (pCR) after NST have significantly improved long-term survival when compared to those did not [3,4].

Taxanes are essential in the adjuvant treatment of lymph-node-positive or high-risk, lymph-node-negative breast cancer [5], and also significantly increased clinical response and pCR rates for operable breast cancer in the neoadjuvant setting [6]. Paclitaxel is one of the most widely used taxanes in breast cancer treatment. Neoadjuvant paclitaxel significantly increased tumor response, and improved survival outcome in those patients who achieved pCR [7–13]. However, paclitaxel contains a combination of polyethylated castor oil and ethanol as the solvents to increase drug solubility, which causes solvent-related toxicities such as hypersensitivity reactions and prolonged peripheral neuropathy [14, 15]. Clinically, paclitaxel should be administered with steroid and antihistamine prophylaxis over a prolonged period of time (3 hours).

Nanoparticle albumin-bound paclitaxel (nab-paclitaxel) is a novel nanometersized particle initially developed to avoid the toxicities associated with polyethylated castor oil [16]. It has been hypothesized that albumin-mediated delivery may result in enhanced transport of nab-paclitaxel to tumors [17] and improved tolerability profile of nab-paclitaxel compared with that of paclitaxel at equimolar doses, with shorter infusion schedules (30 minutes) and no premedication [16]. In a pivotal phase III trial of patients with metastatic breast cancer(MBC), nab-paclitaxel at a dose of 260 mg/m^2^ has been shown to achieve higher response rates and longer time to progression compared to paclitaxel 175 mg/m^2^ (both given every 3 weeks) [18]. The safety profiles of nab-paclitaxel were acceptable in most early trials [19–21], but the data of head-to-head comparison between nab-paclitaxel and paclitaxel is still lacking.

However, in a curative breast cancer setting, no data is available on whether nab-paclitaxel is equivalent or even superior to conventional taxanes (paclitaxel, docetaxel). Several neoadjuvant clinical trials investigated safety and efficacy of nab-paclitaxel-based regimens in operable/locally advanced breast cancer patients. It was hard to interpret all the information into a clear conclusion in terms of the value of nab-paclitaxel in neoadjuvant setting due to: 1) Most of the studies were single-arm, non-randomized phase II trials with rather small sample size, 2) disease subtypes varied among studies, 3) variable study designs regarding to different dose, schedule, drug combination of nab-paclitaxel, 4) different definitions of pCR. Therefore, by reviewing all the neoadjuvant nab-paclitaxel-related studies to date, we performed this meta-analysis with the aim to 1) assess the efficacy of nab-paclitaxel in unselected patients as well as in various intrinsic breast cancer subtypes with specific pCR definitions, 2) to compare efficacy and toxicity of nab-paclitaxel to conventional taxane regimens in neoadjuvant breast cancer treatment.

## RESULTS

### Literature search results

Our literature search yielded 184 relevant records. Twenty-one studies (11 articles and 10 conference abstracts), including 2357 patients who had been treated with neoadjuvant nab-paclitaxel, met the inclusion criteria and were eventually selected for meta-analysis (Figure 1). Eligible trials enrolled patients between 2010 and 2016.

**Figure 1:** The flow chart summarizing the process for the identification of the eligible studies

### Trial characteristics and treatment details

Main characteristics of included trials were listed in Table 1. Twenty studies reported pCR outcomes with the definition of ypT0/is ypN0 (absence of residual invasive cancer within both the breast and lymph nodes, noninvasive breast residuals allowed), while 6 using ypT0/is ypN0/+ (absence of invasive breast cancer in the breast only) and 2 using ypT0 ypN0 (complete eradication of all invasive and noninvasive cancer), respectively. Subgroup analysis according to disease subtypes was conducted in studies whose pCR defined as ypT0/is ypN0. Three randomized studies [43, 47, 48] comparing efficacy of nab-paclitaxel to conventional taxane regimens (paclitaxel or docetaxel) were included in our meta-analysis. Toxicity analyses were also performed within randomized controlled trials [47, 48].

**Table 1:** Baseline characteristics of the included studies

Study	Year	Phase	N	Population	Stage	Neoadjuvant Regimens	Nab-paclitaxel dosage	Definition of pCR	pCR rate(%)
Robidoux[22]	2010	II	65	all	IIB-IIIB	nab-P(H)→FEC(H)	100mg, qw*12	ypT0/is ypN0 ypT0/is ypN0/+	26.2 29.2
Yardley[23]	2010	II	116	all	II-III	nab-P+Gem+E	175mg, q2w*6	ypT0 ypN0	19.8
Sinclair[24]	2012	II	55	HER2-	II-III	nab-P+Cb+bev(→ddAC+bev)	100mg, qw*12	ypT0/is ypN0	34.5
Li[25]	2012	II	54	all	II-III	ddAC(H)→nab-P+Cb(H)	100mg, d1,8,15, q4w*3	ypT0/is ypN0	27.8
Snider[26]	2013	II	30	TN	≥2cm	nab-P+Cb+bev→AC+bev	100mg, d1,8,15, q4w*4	ypT0/is ypN0 ypT0/is ypN0/+	53.3 56.7
Sinclair[27]	2013	II	53	HER2+	II-III	nab-P→Cb	100mg, qw*18	ypT0/is ypN0	45.3
Mrozek[28]	2014	II	33	HER2-	II-III	nab-P+Cb+bev	100mg, d1,8,15, q4w*6	ypT0/is ypN0	18.2
Shimada[29]	2015	NR	53	HER2-	II-III	nab-P→EC	260mg, q3w*4	ypT0/is ypN0 ypT0/is ypN0/+	3.8 5.7
Connolly[30]	2015	II	62	HER2-, Grade 2/3	T1c, N1–3 or T2–4, any N,	nab-P+Cb+/-vorinostat	100mg, qw*12	ypT0/is ypN0	27.4
Huang[31]	2015	II	30	all	II-III	nab-P+Cb(H)	125mg, qw*12	ypT0/is ypN0	26.7
Tanaka[32]	2015	II	45	HER2+	I-IIIA	EC/FEC→nab-P+H	260mg, q3w*4	ypT0/is ypN0	48.9
Gluz[33]	2015	II	324	TN	T1c-T4, any N	nab-P+Cb/Gem	125mg, d1,8, q3w*3	ypT0/is ypN0	36.4
Kuwayama[34]	2015	II	75	HER2-	II-III	nab-P→FEC	100mg, d1,8,15, q4w*4	ypT0/is ypN0	17.3
			77			T→FEC		ypT0/is ypN0	11.7
Khan[35]	2015	II	32	HER2-	II-III	nab-P+H→AC	100mg, qw*12	ypT0/is ypN0	21.9
Shigematsu[36]	2015	II	54	all	T1c-3N0-2	nab-P+C(H)→FEC	260mg, q3w*4	ypT0/is ypN0 ypT0/is ypN0/+	37.0 38.9
Somlo[37]	2015	NR	38	TN	II-III	nab-P+Cb	80mg, qw*16	ypT0/is ypN0	52.6
Untch[38]	2016	III	606	all	>2cm or 1-2cm and high risk	nab-P(H+Per) →EC(H+Per)	150-125mg, qw*12	ypT0/is ypN0 ypT0/is ypN0/+ ypT0 ypN0	42.7 48.7 38.4
			600			P(H+Per) →EC(H+Per)		ypT0/is ypN0 ypT0/is ypN0/+ ypT0 ypN0	34.5 39.7 29.0
Gianni[39]	2016	III	346	HER2- (Luminal-B or TN)	T2-4, N0-3	nab-P→A(E)C/FEC	125mg, d1,8,15, q4w*4	ypT0/is ypN0	22.5
			349			P→A(E)C/FEC		ypT0/is ypN0	18.6
Matsuda[40]	2016	II	35	HER2-	NR	panitumumab→panitumumab +nab-P+Cb→FEC	100mg, d1,8,15, q4w*4	ypT0/is ypN0	28.6
Khasraw[41]	2016	NR	40	all	II-III	EC→nab-P(H)	125mg, d1,8,15, q4w*4	ypT0/is ypN0 ypT0/is ypN0/+	47.5 55.0
Nahleh[42]	2016	II	211	HER2-	IIB-IIIC	nab-P(+/-bev) →ddAC	100mg, qw*12	ypT0/is ypN0	28.0

Abbreviations: nab-P, nab-paclitaxel; pCR, pathologic complete response; NR, not reported; HER2, human epidermal growth factor receptor 2; TN, triple negative; qw, once weekly; q2w, every 2 weeks; q3w, every 3 weeks; q4w, every 4 weeks; H, trastuzumab; FEC, fluorouracil/epirubicin/cyclophosphamide; Cb, carboplatin; bev, bevacizumab; dd, dose dense; AC, doxorubicin/cyclophosphamide; EC, epirubicin/cyclophosphamide; Gem, gemcitabine; T, docetaxel; Per, pertuzumab; P, paclitaxel; ypT0/is ypN0, absence of invasive cancer in the breast and axillary nodes; ypT0/is ypN0/+, absence of invasive cancer in the breast, irrespective of nodal involvement; ypT0 ypN0, absence of invasive cancer and in situ cancer in the breast and axillary nodes.

### pCR after neoadjuvant nab-paclitaxel in unselected population

Overall frequency of pCR was quite satisfying in unselected breast cancer patients treated with neoadjuvant nab-paclitaxel-based regimens. pCR (ypT0/is ypN0) rates ranged between 4% and 53%, with a pooled rate of 32% (95% CI 25-38%) (Figure 2A). The frequency shifted with the stringency of pCR definitions: 29% (95% CI 11-48%) achieved ypT0 ypN0 (Figure 2B), and 39% (95% CI 19-58%) achieved ypT0/is (Figure 2C). ypT0/is ypN0 definition was used in the following analysis.

**Figure 2:** Forest plots of probability achieving pCR in unselected breast cancer patients with pCR definition of (A) ypT0/isN0; (B) ypT0N0; (C) ypT0/is

### pCR in subgroup analyses

As expected, frequency of pCR in patients with hormone receptor positive, human epidermal growth factor receptor 2 negative(HR+/HER2-) tumors was low (14%, 95% CI 11-17%) (Figure 3A). The more aggressive subtypes triple negative breast cancer (TNBC) (41%, 95% CI 38-45%) and HER2+ tumors (54%, 95% CI 43-66%), had increased frequencies of pCR (Figure 3B, 3C). Within the HER2+ population, pCR was more common for HR- tumors (61%, 95% CI 47-74%) than for HR+ tumors (40%, 95% CI 28-52%) (Figure 3D, 3E).

**Figure 3:** Forest plots of probability achieving pCR(ypT0/isN0) in (A) HR+/HER2- group; (B) TNBC group; (C)HER2+ group; (D) HR+/HER2+ group; (E) HR-/HER2+ group

### Efficacy comparison in randomized trials

Three randomized trials, including 2,053 breast cancer patients, compared neoadjuvant nab-paclitaxel versus conventional taxane (paclitaxel/docetaxel). Patients with HER2+ disease in GeparSepto trial were also treated with trastuzumab and pertuzumab, while the other two trials both included only HER2- patients. The schedules and dosages of nab-paclitaxel in each study were as below: in GeparSepto trial, patients received nab-paclitaxel 125 mg/m^2^ continuous weekly for 12 weeks (reduced from the initial dose of 150 mg/m^2^ after a protocol amendment due to high frequency of grade 3-4 peripheral sensory neuropathy) followed by epirubicin/cyclophosphamide(EC); in ETNA trial, a lower dose of nab-paclitaxel 125 mg/m^2^ in 3 out of 4 weeks for 4 cycles followed by EC; and 4 cycles of nab-paclitaxel 100 mg/m^2^ every 3 out of 4 weeks followed by 4 cycles of epirubicin,5-fluorouracil and cyclophosphamide. In the control group, taxane regimens were all given at a standard dose or beyond: in GeparSepto trial, patients were administrated with paclitaxel 80 mg/m^2^ continuous weekly for 12 weeks followed by EC; 4 cycles of paclitaxel 90mg/m^2^ every 3 out of 4 weeks followed by EC were given in ETNA trial; 4 cycles of docetaxel 75 mg/m^2^, every 3-week were given in Kuwayama study. When compared to conventional taxane regimens, patients with neoadjuvant nab-paclitaxel achieved significantly more frequent pCR (OR = 1.383, 95%CI 1.141-1.676, *p* = 0.001) (Figure 4A). A funnel plot of the effect size for each randomized trial against the precision showed no asymmetry (Figure 4B), which indicating no potential publication bias.

**Figure 4:** **A.** Forest plots of odds ratios for pCR within randomized clinical trials. **B.** Funnel plot

### Toxicity profiles

Most nab-paclitaxel trials included in our study demonstrated reasonable tolerability profiles. Safety data from randomized GeparSepto and ETNA trial was extracted to compare the toxicity profiles of nab-paclitaxel to paclitaxel in the preoperative setting. One thousand eight hundreds and seventy eight patients were eventually included into safety analysis, the numbers of all adverse events and those worse than grade 3 were listed in Table 2.

**Table 2:** Safety analysis of nab-paclitaxel compared to paclitaxel (total N=1878)

Toxicity	No. of events		OR	95%CI	P value	Heterogeneity χ^2^	Heterogeneity p value	I^2^(%)
	Nab-paclitaxel	Paclitaxel						
Neutropenia								
Any grade	672	609	1.449	1.162∼1.809	0.001	1.65	0.199	39.3
Grade ≥3	471	437	1.294	0.704∼2.381	0.407	8.28	0.004	87.9
Leucopenia								
Any grade	642	619	1.213	0.916∼1.607	0.178	0.60	0.438	0
Grade ≥3	308	295	1.066	0.863∼1.315	0.554	0.13	0.718	0
Increased alanine aminotransferase								
Any grade	364	379	0.907	0.737∼1.116	0.356	1.73	0.188	42.3
Grade ≥3	16	17	0.655	0.114∼3.744	0.634	2.56	0.109	61.0
Increased aspartate aminotransferase								
Any grade	250	235	1.089	0.873∼1.357	0.451	1.01	0.315	0.9
Grade ≥3	6	6	0.994	0.334∼2.958	0.991	1.48	0.224	32.5
Peripheral sensory neuropathy								
Any grade	725	572	2.090	1.016∼4.302	0.045	12.07	0.001	91.7
Grade ≥3	78	22	3.766	2.324∼6.100	<0.001	0.81	0.369	0
Nausea								
Any grade	615	612	0.995	0.821∼1.206	0.963	0.02	0.900	0
Grade ≥3	28	27	1.031	0.603∼1.764	0.910	0.16	0.691	0
Fatigue								
Any grade	616	561	1.337	1.084∼1.648	0.007	0.15	0.703	0
Grade ≥3	38	29	1.316	0.804∼2.156	0.275	0.58	0.446	0
Vomiting								
Any grade	228	206	1.132	0.913∼1.403	0.259	1.17	0.280	14.3
Grade ≥3	21	18	1.163	0.615∼2.199	0.641	1.97	0.160	49.3
Diarrhea								
Any grade	388	345	1.174	0.877∼1.571	0.282	2.00	0.157	50.1
Grade ≥3	27	20	1.352	0.752∼2.430	0.313	0.81	0.369	0
Rash								
Any grade	249	188	1.347	0.890∼2.038	0.159	2.76	0.097	63.7
Grade ≥3	7	7	0.710	0.063∼7.992	0.782	2.47	0.116	59.5
Hypersensitivity								
Any grade	107	145	0.517	0.201∼1.329	0.171	3.96	0.047	74.8
Grade ≥3	4	7	0.566	0.165∼1.940	0.365	0.02	0.899	0

The hematological toxic effects, neutropenia, leucopenia, increase of alanine aminotransferase, increase of aspartate aminotransferase were generally equivalent but numerically higher in nab-paclitaxel group than paclitaxel group. For non-hematological toxic effect, all grades of peripheral sensory neuropathy occurred more frequently in nab-paclitaxel group as compared to paclitaxel group(OR = 2.090, 95%CI 1.016-4.302, *p* = 0.045). Patients received nab-paclitaxel were 3 times more likely to have severer than grade 3 peripheral sensory neuropathy events (OR = 3.766, 95%CI 2.324-6.100, *p* < 0.001). Hypersensitivity was more common with paclitaxel than nab-paclitaxel at any grade and at grades 3-4, even though that patients in the paclitaxel group already received premedication. Other non-hematological toxic effects, such as nausea, vomiting, fatigue and diarrhea at any grade were identical in two groups.

## DISCUSSION

In this systematic review and meta-analysis, we demonstrate that nab-paclitaxel is an effective cytotoxic drug as in neoadjuvant chemotherapy for primary breast cancer patients, especially in aggressive subtypes. Moreover, this is the first meta-analysis of randomized clinical trials in breast cancer, indicating neoadjuvant nab-paclitaxel significantly improved pCR rate compared to conventional taxanes with generally reasonable toxicity profiles.

In our study, nab-paclitaxel among unselected primary breast cancer patients showed a wide range of pCR rates from 4% to 53%, with a fairly high overall rate of 32%. It is higher than the pCR rate (ypT0/is N0, 19.8%), reported in the German Breast Group (GBG) pooled analysis including seven prospective clinical trials using neoadjuvant anthracycline plus conventional taxane chemotherapy [43]. Additionally, nab-paclitaxel has shown promising early response in neoadjuvant setting. The latest results of ETNA trial showed a clinical overall response rate of 69.4% after first 4 cycles of single-agent neoadjuvant nab-paclitaxel, even though the improved pCR rate with nab-paclitaxel did not reach statistical significance [39]. In WSG-ADAPT TN trial, significant tumor necrosis in 3-week re-biopsy was detected in 24% of the patients after first cycle of nab-paclitaxel, which could contribute to the prediction of pCR rate [33].

Furthermore, patients with more aggressive tumors seemed to benefit from the exchange of nab-paclitaxel. pCR rates in HR-/HER2+ group (61%, 95% CI 47-74%) and TNBC group (41%, 95% CI 38-45%) were much higher than those observed in other breast cancer subtypes. Patients with HR+/HER2- breast cancer had the lowest incidence of pCR (14%, 95% CI 11-17). Pooled-analysis indicated that pCR was significantly more common in patients treated with neoadjuvant nab-paclitaxel when compared to conventional, standard dose or beyond taxanes (OR = 1.383, 95%CI 1.141-1.676, *p* = 0.001). Of note, in the GeparSepto trial, pCR rate almost doubled in the TNBC cohort treated with nab-paclitaxel compared to paclitaxel [38]. Similarly, TNBC patients treated with first-line nab-paclitaxel in metastatic setting also achieved excellent tumor response [44, 45]. Therefore, nab-paclitaxel might be a reasonable taxane-based regimen for curable TNBC patients due to lack of promising ways to further improve the outcomes, but future study is warranted.

In order to improve the benefit of systemic treatment, predictive biomarkers are important in tailoring individualized anti-cancer therapy. But so far we have failed to identify any subset most likely to benefit from neoadjuvant nab-paclitaxel. Secreted protein acidic and rich in cysteine (SPARC) is an albumin and calcium binding glycoprotein, one of its main function is to facilitate tissue remodeling [46]. Hypothetically, an accumulation of SPARC in breast cancer cells and stroma could increase its ability to bind albumin, therefore might serve as a predictive marker for nab-paclitaxel. In the GeparTrio trial, investigators found that high expression of SPARC in tumor cells was significantly correlated with increased pCR rate to neoadjuvant chemotherapy [47]. However, in the GeparSepto trial, the benefit difference from neoadjuvant nab-paclitaxel in the SPARC-overexpressing group was not remarkable compared to the SPARC-negative cohort [38]. Data in metastatic setting also failed to prove association between efficacy of nab-paclitaxel and SPARC expression [48]. More evidences from large prospective trials are warranted to find predictive markers for nab-paclitaxel treatment.

In this meta-analysis, nab-paclitaxel has almost identical toxicities as conventional taxanes except peripheral sensory neuropathy. Both any grade and grade 3-4 peripheral sensory neuropathy were significantly more frequent in nab-paclitaxel group compared to the conventional taxane group. In GeparSepto trial, after dose amendment of nab-paclitaxel from 150 to 125 mg/m^2^ continuous weekly for 12 weeks, the frequency of grade 3-4 peripheral sensory neuropathy in nab-paclitaxel group decreased from 15% to 8% [38]; in ETNA trial, when nab-paclitaxel was given 125 mg/m^2^ every 3 out of 4 weeks for 4 cycles, the frequency of grade 3-4 peripheral sensory neuropathy was 4.5%, which might be one of the explanations that the primary endpoint of this trial, improved pCR after nab-paclitaxel, did not meet statistical significance [39]. Long-term follow-up would be necessary to identify symptom relief patterns and its impact on quality of life.

Notably, in our analysis, patients had less hypersensitivity events in nab-paclitaxel group even though premedication was already given in the conventional group. A few clinical-economic studies supported the cost-effectiveness of nab-paclitaxel in MBC when compared to conventional taxanes since it lowered the incidence of severe adverse events and expenses of managing the critical clinical situations [49, 50].

In conclusion, our study demonstrates that nab-paclitaxel is an effective cytotoxic drug in neoadjuvant treatment of breast cancer, especially in patients with aggressive tumors like TNBC and HER2+ diseases. Exchange of neoadjuvant nab-paclitaxel for conventional taxanes could significantly improve the probability of pCR with generally reasonable toxicities.

## MATERIALS AND METHODS

### Study selection

According to the Preferred Reporting Items for Systematic Reviews and Meta-Analyses (PRISMA) guideline [51], a systematic search of Pubmed was performed using the medical subject heading (MeSH) terms “breast neoplasms”, as well as the following keywords: (1) breast cancer; AND (2) nab-paclitaxel OR nanoparticle paclitaxel; AND (3) neoadjuvant OR preoperative OR primary systemic. The “related articles” function was used to broaden the search. All abstracts, studies and citations were checked for additional material when appropriate. In addition, abstracts from annual meetings of the American Society of Clinical Oncology (ASCO), European Society of Medical Oncology Conference (ESMO) and San Antonio Breast Cancer Symposium (SABCS) were retrieved for relevant abstracts using similar search terms. No language restrictions were made but all available comparative studies were in English language.

### Data extraction

Two investigators (Y Zong, JY Wu) independently performed the search, reviewed and extracted the following data from each study according to a pre-specified protocol: first author, year of publication, study demographics, study design, number of subjects, treatment regimen, and end-point data (pCR). Where discrepancies arose, papers were re-examined and consensus was reached by discussion.

### Inclusion and exclusion criteria

Studies included in the analysis had to comply with all of the following criteria:

1. Studies that reported pCR from neoadjuvant nab-paclitaxel-containing regimen in non-metastatic breast cancer patients;

2. Full paper or conference abstract available;

3. Clear definition of pCR (ypT0/is ypN0, ypT0 ypN0, or ypT0/is ypN0/+).

4. More than 30 eligible patients reported.

5. At least 9 dosages of weekly nab-paclitaxel or 3 cycles of every-3-week nab-paclitaxel.

Studies would be excluded by any one of the following criteria:

1. Studies about adjuvant chemotherapy or metastatic breast cancer;

2. pCR not used as end point for treatment response evaluation;

3. Studies lacking key information.

### Outcomes of interest

The primary endpoint of interest in our study was the total number of patients who achieved pCR, the definition of which varied significantly among the studies included. We conducted our analysis according to each definition of pCR, including ypT0/is ypN0, ypT0 ypN0 and ypT0/is ypN0/+, in order to obtain more detailed and precise results. Besides, comparison of the toxicity profiles of nab-paclitaxel and paclitaxel in randomized trials was also performed.

### Statistical analysis

Aggregate pCR rates were calculated in the nab-paclitaxel-containing arm and the no-nab-paclitaxel arm. Dichotomous data for each trial were expressed as an odds ratio (OR), with 95% confidence intervals (CIs). An OR of >1 favors the nab-paclitaxel group, and the point estimate of the OR was considered statistically significant at the P < 0.05 level if the 95% CI did not include the value of one. Statistical heterogeneity was calculated using Cochrane’s Q statistic and quantified using the I^2^ statistic. Pooled estimates of outcomes were calculated using a fixed-effect model (Mantel-Haenszel test) but a random-effect model (DerSimonian-Laird test) was used when heterogeneity was present. The software package STATA (version 14.0, College Station, TX, US) for Windows 10 was used for analysis.
